The article "Spatiotemporal Relationship between Ecosystem Service Value and Ecological Risk in Disaster-Prone Mountainous Areas: Taking the Upper Reaches of the Minjiang River as an Example" was published in 2022. Journal: J Environ Public Health.

# Spatiotemporal Relationship between Ecosystem Service Value and Ecological Risk in Disaster-Prone Mountainous Areas: Taking the Upper Reaches of the Minjiang River as an Example

**DOI:** 10.1155/2022/1462237

**Published:** 2022-10-07

**Authors:** Linsen Duan, Huaiyong Shao, Mingshun Xiang, Hao Wang, Chunjian Wang, Hao Mei, Yuxiang Tan, Xiaofeng Yang

**Affiliations:** ^1^College of Earth Science, Chengdu University of Technology, Chengdu 610059, China; ^2^Research Center for Human Geography of Tibetan Plateau and Its Eastern Slope, Chengdu University of Technology, Chengdu 610059, China; ^3^College of Tourism and Urban-Rural Planning, Chengdu University of Technology, Chengdu 610059, China; ^4^Piesat Information Technology Co., Ltd, Beijing 100195, China

## Abstract

Mountainous areas are susceptible to disasters; the frequent occurrence of disasters drives the changes in ecosystem service value (ESV) and also brings certain ecological risk, which further increases the incidence of disasters. However, few scholars have investigated the spatiotemporal correlation between the ESV of disaster-prone mountainous areas and ecological risk index (ERI) with basin as the unit. This paper aims to clarify the spatial relationship between ESV and ERI under the changes of land use. Taking the upper reaches of the Minjiang River as the study area, the authors collected the land use data of 2000–2020, estimated ESV by the value equivalent factor per unit area method, and constructed the ERI. On this basis, the relationship between ESV and ERI was investigated in details. The results show the following: (1) From 2000 to 2020, the total ESV exhibited a fluctuating upward trend. The spatial distribution of ESV was greatly affected by slope and altitude; an important reason for the rising ESV in the study area is the increase of forest area and water area. (2) The upper reaches of the Minjiang River had a generally low ERI and relatively good overall ecoenvironment. After 2010, however, the ecological risk continued to rise. Most of the strongly high risk areas are areas with frequent human activities, such as low-altitude areas and river banks. (3) There is a spatial correlation and coupling between ESV and ERI in the study area; i.e., the strongly high ESV areas generally had a low ecological risk. The correlation intensified with the elapse of time. The changes in the service value of regional ecosystems driven by unreasonable land use will have a great impact on the ecoenvironment. By clarifying the spatiotemporal relationship between ESV and ERI, this research provides theoretical basis and data support to the formulation of ecoenvironmental restoration and protection plans for the upper reaches of the Minjiang River and to the coordinated development between society, economy, and ecoenvironment in the region.

## 1. Introduction

Ecosystem service assessment and ecological risk assessment are closely correlated with each other. Both are important aspects of ecosystem quality assessment [1]. Ecosystem services are the supply of various material products and intangible services obtained by humans from the ecosystem. The ecological risk mirrors the ecoenvironmental situation and reflects the security of regional ecology [2, 3]. The integration of ecosystem services and ecological risks can effectively introduce ecosystem services into ecological risk assessment, making ecosystem assessment more complete [4]. At present, the research on ecosystem services and that on ecological risks have gradually moved closer to each other, forming new research hotspots and directions [5].

Land use, the closest bond between human and nature, refers to the way and state of human utilization of the natural features and functions of land [2, 6–10]. Land use changes are an integral part and a major driver of the variation in regional ecoenvironment. It comprehensively reflects the interaction between multiple factors within the terrestrial ecosystem. The continuous change of land use patterns brings changes to the service functions of regional ecosystem [11]. In recent years, many scholars started to study ecoenvironment from the angle of land use. There is a close relationship between land use and ecosystem services. Different types of land use vary significantly in the value of individual ecosystem services. The changes in land use are often resulted from the combined effects of human activities and natural changes, which in turn affect regional ecosystems [12]. The land use pattern affects the living environment and the distribution of resources, as well as the ecosystem service functions. The difference in ecosystem services stems from the disparity in land [13, 14]. Costanza et al. [15] were the first to determine the calculation theory and method of ecosystem service value (ESV). Xie et al. [14, 16] proposed the ESV equivalence system in the light of the actual situation of China and constructed a dynamic evaluation system for China's territorial ecosystem values based on the value equivalent factor per unit area method. Since then, the ESV theory has been continuously applied to assess the ecosystem service capabilities of watersheds, farmlands, cities, wetlands, etc. [17–20]

With the deepening of research, the ecosystem risk caused by land use changes has piqued more and more interests. The land cover variation induced by land use change alters the structure and function of the ecosystem, which in turn influence a series of ecological processes, such as the air, soil, water cycle, and biology [21]. Land use changes, especially land degradation, will bring a string of ecological risks and worsen ecosystem services. Therefore, how to quantify the ecological risk brought by land use has become the focus of research. Relevant research methods include the relative risk model (RRM) [22], the *R* = *P* × *D* model, and the ecological risk index (ERI) [23]. Many algorithms are emerging in the meantime, such as genetic algorithm, ant colony algorithm, and particle swarm optimization [24]. On this basis, multiple evaluation frameworks have been established for the ecological risk under land use changes, namely, the pressure-state-response (PSR) framework, the risk probability-sensitivity-intensity (PSI) framework, the driver-pressure-state-response (DPSR) framework, and the driver-pressure-state-impact-response (DPSIR) framework. These frameworks were utilized to quantify the land use ecological risk in different regions [25–27].

The above analysis shows that land use variation affects the ESV. Irrational use of land will bring ecological risks of different degrees. The relationship between ecosystem and ecological risk under land use changes has always been a key research problem. However, few scholars have investigated the mountain-plain transition zones, which are fragile ecologically and prone to mountain disasters. The upper reaches of the Minjiang River, a typical mountain-plain transition zone in China, serve as a key ecological barrier of the Chengdu Plain, and directly bear on regional ecological security. According to the existing research results, there is a spatiotemporal correlation between the ESV and ecological risks [1, 4, 5]. Based on this understanding, this paper assumes that the spatiotemporal correlation exists in the upper reaches of the Minjiang River and relies on the value equivalent factor per unit area method to quantify the spatiotemporal evolution of ESV and ERI in the study area, using the data on land use. On this basis, the spatial relationship between ESV and ERI was investigated in details. The research results clarify the ecosystem quality of the upper reaches of the Minjiang River from both ESV and ERI, help to grasp the spatiotemporal relationship between ESV and ERI, provide basic data support to the coordinated promotion of the ecosystem service improvement and comprehensive management of the ecoenvironment in the upper reaches of the Minjiang River, and promote the synergistic development between society, economy, and ecoenvironment in the region.

## 2. Materials and Methods

### 2.1. Study Area

The upper reaches of the Minjiang River belong to the eastern margin of the Qinghai-Tibet Plateau (30.7°N–33.2°N, 102.5°E–104.3°E) (Figure 1). With a drainage area of about 24,783.08 km^2^, this region has a great significance ecologically, for it is the primary ecological barrier and water source of the Chengdu Plain. The terrain of the region is high in the northwest and low in the southeast. The mean elevation surpasses 3,000 m. The region is crisscrossed by river valleys with a height difference of more than 5,000 m. There is a huge elevation difference (2,000–3,000 m) between the ridges and river valleys. The study area has various types of landforms, ranging from plateaus to high mountains. Strong tectonic movements have brought frequent geological disasters to the region. Extremely serious mountain geological disasters have hit the region, namely, the Wenchuan earthquake, and the Maoxian County high landslide. In addition, the ecoenvironment is fragile, and soil erosion is serious. As a plateau alpine monsoon climate zone, the study area features vertically distributed climate belts, as well as cold winters and cool summers. The soil types are mainly alpine meadow soil, brown soil, yellow-brown soil, and cinnamon soil; the vegetation types are mainly coniferous forest, shrub, alpine meadow, subalpine coniferous forest, and dry valley shrub.

### 2.2. Research Data

The land use data come from the Resource and Environment Science and Data Center (http://www.resdc.cn), and its spatial resolution is 30 m × 30 m. Using ArcGIS, the land use types were classified into six categories: farmland, forestland, grassland, water area, construction land, and unused land. The main information source is the remote sensing images shot by Landsat satellites. The data of 2000, 2005, and 2010 were taken from the remote sensing images of Landsat-TM/ETM. The data of 2015 and 2020 were taken from those of Landsat 8. The highly precise data guarantee the reliability of the calculated ESV values in the subsequent analysis. The DEM data were obtained from SRTM (Shuttle Radar Topography Mission) of Resources and Environmental Science and Data Center, with a spatial resolution of 30 × 30 m, an absolute horizontal accuracy ±20 m, and an absolute elevation accuracy ±16 m. The elevation and slope were extracted from the downloaded DEM. The socioeconomic data, namely, crop yield per unit area and sown area of crops, are mainly gathered from *China Statistical Yearbooks* and *Sichuan Provincial Statistical Yearbooks*. The food prices were obtained from http://www.scgrain.com/.

### 2.3. Methods

*ESV*. Ecosystem services refer to the life support products and services obtained directly or indirectly through the structure, process, and function of the ecosystem, which are usually evaluated by market valuation and consumer willingness to pay [5]. Costanza et al. divided the global ecosystem services into 17 different types of services and 16 biomes and calculated the global annual ESV, making the quantitative assessment of ESV a research hot topic. This method has been widely to evaluate the value of various ecosystem services [15]. However, their analysis is unfolded on the global scale. If their method is directly adopted, the ESV of the study area in this research will be estimated with large deviations.

Taking the situation in China as the baseline, Xie et al. [14] formulated the following calculation model of economic value, in reference to Costanza's research and the studies of ecological scholars in China [14, 16]:

(1) $$\begin{array}{c} {VC}_{k}=1/7\overset{n}{\underset{i=1}{\sum }}\frac{m_{i}P_{i}q_{i}}{M},i=\left(1,2\cdots \cdots n\right), \end{array}$$

where *VC*_*k*_ is the economic value of the food production function provided by a unit area of farmland ecosystem (yuan/hm^2^); *i* is the type of crop; *P*_*i*_ is the man price of type *i* crop (yuan/kg); *q*_*i*_ is the per unit area yield of type *i* crop (kg/hm^2^); *m*_*i*_ is the sown area of type *i* crop (hm^2^); *M* is the total sown area of all grain crops.

The ESV in the upper reaches of the Minjiang River can be calculated by:

(2) $$\begin{array}{c} ESV=\sum \left(A_{k}\times {VC}_{k}\right), \end{array}$$

where *ESV* is the total value of ecological services; *A*_*k*_ is the area of the *k*th type of land use.

To eliminate the ESV gap of different types of land use between the study area and China, this paper extracts slope and elevation from the DEM data on the upper reaches of the Minjiang River. Drawing on the socioeconomic data like grain yield per unit area and crop sown area, the economic value equivalent factor per unit area of ESV in the upper reaches of the Minjiang River was solved and corrected as 1,305.45 yuan·hm^−2^. On this basis, the authors derived the ESVs per unit area of different lands in the study area (Table 1).

*ERI*. Ecological risk refers the risk that an ecosystem and its components bear under the disturbance of natural or human activities. It refers to the possible adverse effects of uncertain accidents or disasters on the structure and function of ecosystems in a certain area. Numerous studies have shown a close correlation between land use change and ecological risk and considered land use change the greatest impactor of the ecosystem [5]. Using the area ratio of each land type, the authors constructed the ERI and built the empirical relationship between land use structure and regional ecological risk. The relationship was used to measure the relative magnitude of ecological risk in grid units [23]. The ERI can be calculated by:

(3) $$\begin{array}{c} ERI=\overset{N}{\underset{i=1}{\sum }}\frac{A_{ki}}{A_{k}}W_{i}, \end{array}$$

where *ERI* is the ecological risk index; *A*_*k*_ is the total area of the *k*th sample plot; *A*_*ki*_ is the total area of type *i* land in the *k*th sample plot; *W*_*i*_ is the ecological risk intensity of type *i* land; *N* is the number of types of land use.

Comparing different grid sizes, it was found that a large grid size would sacrifice the coupling effect, and a small grid size would result in data redundancy. Finally, 1 km × 1 km was chosen as the optimal grid size. This paper sets the grid size to 1 km × 1 km, with a total of 24,927 grids. The ERI of each type of land use was determined through literature review, in consultation with experts on land management and ecological risk evaluation [28]. The mean ERI of each grid was solved. Through analytical hierarchy process (AHP), the ecological risk intensity *W_i_* of different types of land use was solved: forest land 0.0427, farmland 0.1916, construction land 0.3934, water area 0.1425, grassland 0.0726, and unused land 0.1572 [28].

*Coupling Coordination Degree (CCD) Model*. The CCD model reflects the interplay and action mechanism, and coordination state among the systems in the study area. It is widely used in ecoenvironmental research. This paper adopts the CCD model to measure the coupling coordination relationship between the ESV and ERI in the upper reaches of the Minjiang River [27, 28]. The CCD can be calculated by:

(4) $$\begin{array}{c} C=\frac{{{ESV}_{i}}^{k}\times {{ERI}_{i}}^{k}}{{\left(\alpha {ESV}_{i}+\beta {ERI}_{i}\right)}^{2k}}, \end{array}$$

(5) $$\begin{array}{c} D=\sqrt{C\times T}, \end{array}$$

(6) $$\begin{array}{c} T=\sqrt{\alpha {ESV}_{i}\times \beta {ERI}_{i}}, \end{array}$$

where *C* is the coupling degree index; *D* is the CCD index; *T* is the composite evaluation index of the two factors; *ERI*_*i*_ is the normalized ERI of the *i*th year; *ESVi* is the normalized ESV of the *i*th year; *α* and *β* are coefficients to be determined. Here, *α* = *β* = 0.5.

Exploratory Spatial Analysis (ESA). The spatial relationship between ESV and ERI in the upper reaches of the Minjiang River can be judged by the global spatial autocorrelation index [29]:

(7) $$\begin{array}{c} EBI=\frac{m}{\sum_{i=1}^{m}\sum_{j=1}^{m}\;}\frac{\sum_{i=1}^{m}\sum_{j=1}^{m}\omega_{ij}R_{i}R_{j}}{\sum_{i=1}^{m}{\left(R_{i}-\bar{R}\right)}^{2}}. \end{array}$$

The EBI reflects whether the spatial values of the object are similar in space. If *EBI* = 0, the two values are randomly distributed. In formula (7), *w*_*ij*_ is the spatial weight; *R* is the mean attribute value; *R*_*i*_ and *R*_*j*_ are the mean of factors *i* and *j*, respectively; *n* is the number of units. If |*Z*| > 1.96, the correlation is significant.

As a decomposed form of Moran's *I*, the local spatial autocorrelation reflects the internal correlation within the study area. The Moran's *I* index was corrected by empirical Bayesian method to obtain the corrected local autocorrelation index EBI:

(8) $$\begin{array}{c} {EBI}_{i}=\left(R_{i}\sqrt{V_{i}}\overset{m}{\underset{j=1}{\sum }}\omega_{ij}\left(R_{ij}\sqrt{V_{i}}\right)\right). \end{array}$$

## 3. Results

### 3.1. Spatiotemporal Evolution Features

The ESVs in the upper reaches of the Minjiang River in 1995–2020 were solved by formula (1), in reference to Table 1. The results are shown in Table 2.

As shown in Table 2, the total ESV of the study area was 4.34 × 10^10^ yuan, 4.33 × 10^10^ yuan, 4.55 × 10^10^ yuan, 4.55 × 10^10^ yuan, and 4.56 × 10^10^ yuan, respectively, in 2000, 2005, 2010, 2015, and 2020. The total value firstly decreased and then gradually increased, but the overall variation was small. The annual mean increase was merely 1.08 × 10^8^ yuan. This is consistent with the conclusion of Xiang et al. [29].

Throughout the research period, the ESV proportion of each land use changed, but the changes did not affect the basic structure of ESV. The proportion of forest land in ESV was always more than 75% in the 25 years. The other types of land had a much smaller ESV than forest land. Hence, forest land is the dominant landscape in the upper reaches of the Minjiang River. Grassland is distributed more widely than any other type of land. However, the ESV per unit area of grassland was far smaller than that of forest land. That is why grassland ranked the second in ESV proportion throughout the study period.

In terms of the spatiotemporal variation in ESV, the ESV of the study area reduced by 2.61 × 10^7^ yuan from 2000 to 2005. The main reason is the decline in the total ESV of forest land. Grassland was the land type with the largest ESV increment (5.72 × 10^4^ yuan), while forest land was the land type with the largest ESV decrement (5.31 × 10^6^ yuan).

From 2005 to 2010, the ESV of the study area saw a net growth of 2.13 × 10^9^ yuan, up by 4.9% from the previous period. The main contributor is the ESV growth (196.82%) of the water area. In this period, forest land also witnessed a rapid growth of total ESV. Both water area and forest land promoted the rapid growth of ESV.

From 2010 to 2020, the ESV of the study area increased rather slowly, up by only 0.14%, with a net increase of 6.56 × 10^5^ yuan. In this period, the water area's ESV continued to increase, realizing a net growth of 1.16 × 10^6^ yuan. On the contrary, the ESV of forest land dropped sharply by 5.03 × 10^5^ yuan.

Although the uncontrolled expansion of farmland was controlled by the grain for green policy, the high ESV forest land shrunk in the period, owing to the complex topography and frequent disasters in the Minjiang River Basin. As a result, the ESV growth driven by the water area was offset by the ESV loss of forest land. Overall, the total ESV of the study area did not change much in the period. These results suggest that the relevant policies in the upper reaches of the Minjiang River benefit ESV increase, but the rapid loss of ESV in local areas calls for more attention.

### 3.2. Spatiotemporal Evolution Features of ERI

The stable model was used to perform ordinary kriging interpolation on the ecological risk values of 24,927 sample areas in the upper reaches of the Minjiang River during the study period, and the ERI was divided into strongly high ecological risk (≥0.20), slightly high ecological risk (0.15–0.20), medium ecological risk (0.10–0.15), slightly low ecological risk (0.05–0.10), and strongly low ecological risk (<0.05). The area of each level was counted by the spatial analysis tool of ArcGIS10.2. The results are shown in Figure 2.

As shown in Figure 2(a), there was a certain difference in the spatial distribution of ERI in the upper reaches of the Minjiang River from 2000 to 2020, but the overall change was not large. Most of the areas were strongly low and slightly low ecological risk areas. The strongly low ecological risk areas were relatively concentrated, while the strongly high and slightly high ecological risk areas were scattered and not connected. On the spatiotemporal variation of ecological risk, the trend of 2000–2005 is dominated by the change of strongly low-risk areas in the center of the study area, that of 2005–2010 is dominated by the change of strongly high risk areas in the north and south of the study area, and that of 2010–2020 is not significant. The slightly high and strongly high risk areas were located in Chuanzhusi Town and Jin'an Town in the north; Luhua Town, Weigu Township, and Seergu Town in the middle; Shunfu Township and Weimen Township in the east; and Xuankou Town and Sanjiang Town in the south. The strongly low ecological risk areas were relatively concentrated, mainly in Gengda Town, Caopo Township, Putou Town, and Puxi Township in the south, and Baiyang Township in the central and eastern part of the basin. The northern and southern margins of the study area were the main distribution areas of slightly low ecological risk areas, mainly involving Chuanzhusi Town, Caoyuan Township, Minjiang Township, Yanyun Township, Yinxing Township, and Wolong Town.

As can be seen from Figure 2(b), it should be noted that from 2020 to 2020, although the strongly low and slightly low ecological risk areas dominated the study area, the slightly low ecological risk areas decreased from 19027.1 to 18374.1 km^2^. Meanwhile, the slightly high and strongly high risk areas in 2020 were 2.5 times and 14 times that in 2000, respectively. Overall, there was a continuous growth of ecological risks in local areas.

### 3.3. Spatial Relationship between ESV and ERI

The spatial coupling index between ESV and ERI was calculated by formula (4). Then, the coupling degree of each year was divided into five levels by the natural breakpoint method. The total area of each coupling degree was summarized by ArcGIS 10.2 (Figure 3).

As shown in Figure 3(a), the coupling degree of ESV and ERI in the upper reaches of the Minjiang River exhibited an obvious spatial differentiation, and the overall coupling degree was low in the north and high in the south. The areas with slightly high coupling degree were the most widely distributed. Such areas were mainly distributed like patches in the river valleys in Wenchuan County and Lixian County and scattered in other places. The slightly low coupling degree was mainly observed in the high-altitude areas; the medium coupling degree was mostly detected along the margins of the areas of strongly high coupling degree. In addition, the strongly high and strongly low coupling degrees were sporadically distributed.

As shown in Figure 3(b), the areas with strongly low or strongly high coupling degree occupied a very small portion of the study area. In the study period, however, both types of areas exhibited a growing trend. The areas of strongly low coupling degree expanded from 171 to 193 km^2^, while those of strongly high coupling degree increased by nearly six times, from 105 to 626 km^2^.

In general, the areas with slightly low, medium, and slightly high coupling degrees shrunk slightly in the study period. The areas with slightly high coupling degree boasted the highest proportion (43%), while the proportions of the areas with slightly low coupling degree and those with medium coupling degree did not change much, which remained at around 29% and 26%, respectively. Judging by the coupling between ERI and ESV, the high ESV areas are coupled closely with the low ERI areas, indicating the spatial correlation between ESV and ecological risk.

Further analysis of the CCD between ESV and ERI in the study area (Figure 4) shows that ERI and ESV were in coordinated development in most areas, but large stretches of uncoordinated development were observed. From 2000 to 2005, the CCD was high in the middle and south, forming patches in the south, and low and scattered in the north. From 2005 to 2020, the CCD in the north was optimized, and the strongly high coordinated areas increased along river valleys. In terms of the type of coupling coordination, the strongly high coordinated areas occupied a small portion, which increased significantly since 2010. The increase was mainly achieved in river valleys of Heishui County, Lixian County, and Wenchuan County. Many strongly uncoordinated areas existed in scattered form from 2000 to 2015. From 2005 to 2020, the strongly uncoordinated areas were generally on the decline.

Spatial Relationship Analysis Based on Autocorrelation Method. The spatial autocorrelation index between ESV and ERI was calculated by formula (7). The results in Figure 5 show that the Moran's *I* between ESV and ERI in the upper reaches of the Minjiang River was 0.018, 0.018, 0.018, 0.025, 0.025, and 0.021, respectively. EBI was always greater than 0, indicating that there was a certain spatial correlation. The overall correlation was not high. The global spatial correlation analysis shows that the spatial distribution of ERI and ESV in the upper reaches of the Minjiang River was not random. There was a certain correlation between ecological risk and ESV, but the relationship was relatively weak. After 2005, the degree of correlation continued to increase. However, the correlation started to weaken in 2020. Therefore, it is necessary to take targeted ecological restoration measures, optimize the ecosystem environment in discrete areas, and continuously enhance the ecosystem service capacity.

Further, the local spatial autocorrelation between ESV and ERI was calculated by formula (8). The results in Figure 6 show that the high-high and low-low cluster areas of ESV and ERI correlation in the study area were basically stable. The high-high cluster areas were scattered in the middle; the low-low areas were mostly concentrated in river valleys; the low-high and high-low areas were rather few. ESV and ERI were uncorrelated in most cases.

When it comes to the time-variation of the spatial correlation between ESV and ERI, after 2005, the high-high areas in the north declined clearly, while those in the south became less concentrated. This trend is closely associated with the grain for green project and mainly affected by human activities. Hence, the high-high areas largely fell to regions with intense human activities.

There were many low-low areas of ESV-ERI correlation, most of which belonged to the south and middle of the study area. A few low-low areas concentrated in the east. Thus, the low ERI areas have a slightly high ESV. The main reason is as follows: this area is mainly an ecological reserve, with a humid and mild climate. After the Wenchuan earthquake, ecological restoration and protection were accelerated, the vegetation coverage was fully restored, and the landscape was no longer fragmented.

## 4. Conclusions and Discussion

This paper targets the main ecoenvironmental problems in the upper reaches of the Minjiang River, a typical mountain-plain transition zone in China, and quantifies the spatiotemporal evaluation features of ESV and ERI in the region, using the land use data, and, on this basis, explores the spatial relationship between the two factors. The main conclusions are as follows:

1. From 2000 to 2020, the total ESV exhibited a fluctuating upward trend; the areas with a slightly high ESV increased with fluctuations and were distributed relatively concentratedly. In most towns and townships in the study area, the ESV belonged to the slightly low and slightly high levels. The spatial distribution of ESV was greatly affected by slope and altitude, which led to obvious differences in its spatial distribution
2. The upper reaches of the Minjiang River had a strongly to slightly low ERI, and a slightly low ERI. The medium, slightly high, and strongly high risk areas took up small proportions in the study area, a sign of relatively good overall ecoenvironment. From 2005 to 2010, the ecological risk changed violently, owing to the Wenchuan earthquake and its secondary disasters. After 2010, slightly high and strongly high risk areas continued to widen. The new slightly high and strongly high risk areas mainly belonged to regions with frequent human activities, such as low altitude areas and river banks
3. In the study area, very few regions had strongly low or strongly high coupling degrees between ESV and ERI, but more and more regions witnessed a strongly high coupling degree. The CCD was mainly strongly low, medium, and strongly high and went through violent spatial changes with the elapse of time. There was a certain spatial correlation between ESV and ERI. The low-low cluster feature was very prominent, suggesting that high ESV areas tend to have a slightly low ERI
4. The research on the spatiotemporal relationship between ESV and ERI can better link human well-being with the sustainable development of the ecoenvironment and provide decision-making basis for regional ecoenvironmental protection and risk management. This paper focuses on the spatiotemporal relationship between ESV and ERI in the upper reaches of the Minjiang River. However, the changes of regional ESV and ERI are the combined results of multiple factors. Admittedly, this study focuses on the temporal and spatial relationship between ESV and ERI. Yet it fails to fully reflect the relationship and influence the mechanism and evolution trend of these two factors. To make up for the gap, the future research will build a more precise and applicable evaluation system, comprehensively evaluate regional ESV and ERI changes under the combined influence of multiple factors, provide inspiration for IPBES global ecosystem service assessment and IPCC AR6, and contribute more to the control of global warming

## Figures and Tables

**Figure 1:** Location of study area.

**Figure 2:** Spatiotemporal distribution of ecological risks and the area statistics of each ecological risk level.

**Figure 3:** Coupling relationship between ESV and ERI and total area of each coupling degree.

**Figure 4:** CCD between ERI and ESV.

**Figure 5:** Scatterplot of Moran's *I*.

**Figure 6:** Scatterplot of local spatial autocorrelation.

**Table 1:** Ecological value coefficients of various land use types in the upper reaches of the Minjiang River (yuan/hm^2^).

Primary type	Secondary type	Farmland	Forest land	Grassland	Water area	Construction land	Unused land
Supply services	Food production	1109.63	404.69	130.55	1044.36	0.00	0.00
	Raw material production	522.18	926.87	182.76	300.25	0.00	0.00
	Water conservation	26.11	483.02	104.44	10822.18	0.00	104.85

Regulation services	Air regulation	874.65	3067.81	665.78	1005.20	0.00	33.88
	Climate regulation	469.96	9177.31	1749.30	2989.48	0.00	26.21
	Waste disposal	130.55	2597.85	574.40	7245.25	0.00	133.46
	Hydrological regulation	352.47	4582.13	1279.34	133469.21	0.00	383.80

Support services	Soil conservation	1344.61	3733.59	809.38	1214.07	0.00	25.14
	Nutrient recycling maintenance	156.65	287.20	65.27	91.38	0.00	0.00
	Biodiversity conservation	169.71	3394.17	731.05	3328.90	0.00	25.62

Cultural services	Entertainment culture	78.33	1488.21	326.36	2467.30	0.00	16.94

**Table 2:** ESVs in 2000–2020.

Time (year)	Statistical type	Farmland	Forest land	Grassland	Water area	Construction land	Unused land	Sum
2000	Value (10^8^ yuan/year)	3.5264	339.2511	84.6721	6.5496	0.0000	0.0081	434.0073
	Proportion (%)	0.8125	78.1671	19.5094	1.5091	0.0000	0.0019	100

2005	Value (10^8^ yuan/year)	3.5135	338.8580	84.7706	6.5965	0.0000	0.0081	433.7467
	Proportion (%)	0.8100	78.1235	19.5438	1.5208	0.0000	0.0019	100

2010	Value (10^8^ yuan/year)	3.6680	350.5846	81.1639	19.5797	0.0000	0.0233	455.0195
	Proportion (%)	0.8061	77.0482	17.8374	4.2030	0.0000	0.0051	100

2015	Value (10^8^ yuan/year)	3.6336	350.4870	81.1593	19.3758	0.0000	0.0233	454.6789
	Proportion (%)	0.7992	77.0845	17.8498	4.2614	0.0000	0.0051	100

2020	Value (10^8^ yuan/year)	3.6332	350.0814	81.1945	20.7425	0.0000	0.0235	455.6751
	Proportion (%)	0.7973	76.8270	17.8185	4.5520	0.0000	0.0052	100

## Data Availability

The data used to support the findings of this study are available from the corresponding author upon request.
